# Significant Asymmetry of the Bilateral Upper Extremities of a Skeleton Excavated from the Mashiki-Azamabaru Site, Okinawa Island, Japan

**DOI:** 10.1155/2021/4884760

**Published:** 2021-11-17

**Authors:** Keiko Ogami-Takamura, Kazunobu Saiki, Keita Nishi, Tetsuaki Wakebe, Daisuke Endo, Kiyohito Murai, Yoshiatsu Naito, Toshiyuki Tsurumoto

**Affiliations:** ^1^Department of Macroscopic Anatomy, Graduate School of Biomedical Sciences, Nagasaki University, 1-12-4 Sakamoto, Nagasaki, Nagasaki 852-8523, Japan; ^2^Center of Cadaver Surgical Training, School of Medicine, Nagasaki University, 1-12-4 Sakamoto, Nagasaki, Nagasaki 852-8523, Japan; ^3^Department of Anesthesiology and Intensive Care Medicine, Graduate School of Biomedical Sciences, Nagasaki University, 1-7-1 Sakamoto, Nagasaki, Nagasaki 852-8501, Japan; ^4^Department of Oral Anatomy and Dental Anthropology, Graduate School of Biomedical Sciences, Nagasaki University, 1-7-1 Sakamoto, Nagasaki, Nagasaki 852-8588, Japan; ^5^Nagasaki Medical College, 36-59 Atago, Nagasaki, Nagasaki 850-0822, Japan; ^6^Nagasaki University, 1-12-4 Sakamoto, Nagasaki, Nagasaki 852-8523, Japan

## Abstract

The human skeleton of a young adult male with marked asymmetry of the bilateral upper extremities was excavated from the Mashiki-Azamabaru site (3000–2000 BCE) on the main island of Okinawa in the southwestern archipelago of Japan. The skeleton was buried alone in a corner of the cemetery. In this study, morphological and radiographic observations were made on this skeleton, and the pathogenesis of the bone growth disorder observed in the left upper limb was discussed. The maximum diameter of the midshaft of the humerus was 13.8 mm on the left and 21.2 mm on the right. The long bones comprising the left upper extremity lost the structure of the muscle attachments except for the deltoid tubercle of the humerus. The bone morphology of the right upper extremity and the bilateral lower extremities was maintained and was close to the mean value of females from the Ohtomo site in northwestern Kyushu, Japan, during the Yayoi period. It is assumed that the anomalous bone morphology confined to the left upper extremity was secondary to the prolonged loss of function of the muscles attached to left extremity bones. In this case, birth palsy, brachial plexus injury in childhood, and acute grey matter myelitis were diagnosed. It was suggested that this person had survived into young adulthood with severe paralysis of the left upper extremity due to injury or disease at an early age.

## 1. Introduction

The presence of continuous external mechanical stimulation is essential for the maintenance of bone morphology and strength [1, 2]. Persistent paralysis of the motor nerves leads to paralysis of the corresponding muscles and restriction of bone and joint movement. This leads to a decrease in bone strength and subsequent changes in bone morphology. In this study, we present a clinical and social differential diagnosis of a male human skeleton (Mashiki 15) with marked asymmetry of both upper extremities, excavated from the Mashiki-Azamabaru site on the main island of Okinawa, in the southwestern archipelago of Japan in East Asia. According to the archaeological findings, it is considered that the site was constructed in the period 3000–2000 BCE. In the field of palaeopathology, there are not many reports of cases of bilateral asymmetry confined to the upper extremities. It would be of great palaeopathological value to discuss the significant bone asymmetry confined to the upper extremities observed in this case.

## 2. Materials and Methods

The Japanese archipelago is located east of the Asian continent and extends for about 3,500 km in a long, narrow line from north to south. The Ryukyu Islands, to which Okinawa Island belongs, where the Mashiki-Azamabaru site is located, are at the southern end of the Japanese archipelago (Figure 1). This site was discovered in 1981 during the redevelopment of the Mashiki area of Ginowan, Okinawa Prefecture, Japan, and excavations were carried out from 1985 to 1989 [3]. The period of this site is the middle period of the prehistoric shell midden culture on Okinawa Island (3000–2000 BCE). This corresponds to the Late Jomon to early Yayoi periods in Japan. The site is located on a dune in an alluvial lowland 4 to 5 m above sea level, about 180 m from the coastline, and 58 human skeletal remains (51 adults and 7 nonadults) were excavated. Among these human skeletal remains, one human skeleton (Mashiki 15) was found to have significant upper extremity asymmetry, with the left side thinner than the right.

Mashiki 15, discussed in this research, was excavated from the west side of the collective graves and was buried supine and extended in the east-southeast head position (Figure 2). Mashiki 15 was buried alone in a hole-shaped grave, so it is not possible to be confused with other human skeletal remains. The remaining part of Mashiki 15 is shown in Figure 3. The skeletal remains of Mashiki 15 have been legally preserved at our laboratory, which was involved in the excavation project. We investigated Mashiki 15 in detail using standard macroscopic techniques in bioarchaeology [4]. The sex of Mashiki 15 was determined from the morphological features of the skull and pelvic bones. The age of Mashiki 15 was estimated to be young adult based on the degree of closure of the skull's sutures [5] and the degree of occlusion of the crown of the teeth [6]. The estimated height of Mashiki 15 was 165.4 cm by applying Pearson's formula [7] to the maximum length of the right radius, 243 mm. The asymmetry of the extremity bone measurements was examined using the method of Trinkaus et al. [8] and Lieverse et al. [9]: 100 × (maximum − minimum)/minimum. The measurements of Mashiki 15 were compared with the mean values of adult male and female bones and measurements of nonadults (two equivalent to a 9-year-old and one equivalent to a 10-year-old) excavated from the Ohtomo site (Karatsu, Saga Prefecture, Japan; early to mid-Yayoi period, 3000–2000 BCE) in northwestern Kyushu, Japan [10, 11].

Bilateral humerus, radius, and ulna were imaged with a clinical multislice computed tomography (CT) (Activision 16, Toshiba, Tokyo, Japan) (X tube volume/current = 120 kV/100 mA, 0.5 mm thickness). The clinical multislice CT belongs to the Graduate School of Biomedical Sciences, Nagasaki University. Based on the obtained DICOM data, the left and right horizontal morphologies were compared in horizontal cross-sectional images obtained at the midheight of the radius and at the height of the distal quarter of the ulna. The left and right sides of the humerus, radius, and ulna were also compared on horizontal cross-sectional images obtained at the level of the minimum circumference of the diaphysis, measured grossly. All DICOM images were read by two physicians, including a board-certified specialist of the Japanese Orthopaedic Association.

## 3. Results

### 3.1. Skull

The skull remained with the cranial crown, the right side of the face, and the left side around the orbit. There is no pronounced asymmetry in the remaining parts (Figure 4). The maximum cranial length and breadth of the head were 176 mm and 135 mm, respectively, and the maximum cranial breadth was slightly smaller than those of human skeletal remains excavated from the Gushikawajima site (Shimajiri, Okinawa Prefecture, Japan), 173 mm and 145 mm, respectively, which are close to those of the period [12]. The cephalic index was 76.7, indicating mesocephalic. The supraocular height was 65 mm, and although the facial height index cannot be determined from the remaining portion, it suggests a low face. Based on the development of the mastoid process, the protrusion of the marginal tubercle, and the large width of the frontal process, it was assumed to be male. An osteoma was found in the remaining right external auditory canal (Figure 4). The coronal, sagittal, and lambda sutures of the skull were open on the inner and outer plates. The degree of occlusal wear on the crown surface was 1–2 degrees according to Broca's evaluation method [13] and D by Lovejoy's method of evaluation [6], which provided a basis for determining that Mashiki 15 was a young adult.

### 3.2. Lower Extremity

As shown in Figure 3, the distal articular end was missing, but the femur, tibia, and fibula diaphysis were well preserved (Figure 5(a)). The right and left iliacs and part of the sciatic bones were present in the pelvis (Figures 3 and 5(a)). The narrow angle of the bilateral greater sciatic notches provided the basis for determining that this skeleton was male [14].

### 3.3. Upper Extremity

The right carpals remained with the trapezium, trapezoid, scaphoid, capitate, lunate, and triquetrum. Of the right phalanges, all the metacarpals and proximal phalanges and part of the middle phalanges remained. The left carpals and phalanges were not retained. The long bones of the upper extremity remained, the right and left humeri, radius, and ulna. The proximal articular end of the right humerus and the distal articular end of the right ulna were absent. The left humerus, ulna, and radius were absent at both articular ends. The transverse and circumferential diameters of all long bones of the left upper extremity were smaller than those of the right side (Figure 5(b), Table 1). The percentage asymmetry of the humerus was 53.6% for maximum diameter of the midshaft (Martin number; M5), 31.7% for minimum diameter of midshaft (M6), and 40.5% for the least circumference of the shaft (M7). In the radius, the maximum transverse shaft diameter (M4) was 27.0%, minimum sagittal shaft diameter (M5) was 46.6%, and minimum circumference (M3) was 35.7%. In the ulna, the dorsoventral shaft diameter (M11) was 60.7%, transverse shaft diameter (M12) was 75.8%, and least circumference (M3) was 46.2% (Table 1).

The length of the long bones of the left upper extremity was estimated from the remaining parts. The growth in the long axial direction was considered relatively normal. In the long bones of the left upper extremity, the features characteristic of muscle insertion, such as tubercles, tuberosity, crest, and grooves, were almost absent except for the deltoid tuberosity of the humerus (Figure 6(a)). In addition, the diaphyses were thin and had lost their biomechanical structure due to significant inhibition of their diaphyseal maturation. The right radius was preserved to the epiphysis, and this maximum length of 243 mm was applied to Pearson's formula to obtain an estimated height of 162.8 cm. This height is higher than the mean height of 156.8 cm for the male human remains examined at the Gushikawajima site [12] in the Late Jomon period, which is geographically close to the Mashiki-Azamabaru site. As shown in Table 2, the measurements of the left humerus, radius, and ulna of Mashiki 15 were closer to those of a 9-year-old equivalent child than the means of adult males and females at the Ohtomo site [11]. The bone measurements of the right upper extremity of Mashiki 15 were closer to the means of the Ohtomo females [10].

As shown in Table 1, the overall transverse size of the humerus was significantly smaller on the left side. In the radius, the left radial tuberosity was lost post mortem. Therefore, it was not possible to identify any difference between the left and right sides at the articular end. In the radius diaphysis, the interosseous border of the left radius was slightly undeveloped compared to that of the right side (Figure 6(b)).

The left tuberosity of the ulna and the supinator crest were weakly developed and smooth. The interosseous border and posterior border were not well developed. The formation of the interosseous and posterior borders was significantly weaker than the right (Figure 6(c)).

The lateral portion of the clavicle remained on both sides. Although the left side was slightly narrower, there was no difference between the other upper extremity bones.

### 3.4. Computed Tomography Images

Cross-sectional CT images of the left and right humeri, ulna, and radius at the height of the minimum circumference measurement are shown (Figures 7(a)–7(c)). The shapes of the cross-sections of the diaphysis of the humerus, radius, and ulna were distorted and circular. The left and right sides were compared in a slice where the minimum circumference was measured. Although it is difficult to quantitatively assess the cortical bone due to artefacts and defects, a comparison of the images showed cortical bone thinning in the humerus and ulna on the left side compared to the right side. No thinning of the cortical bone was observed for the radius, but the interosseous margin was dulled.

## 4. Discussion

### 4.1. The Process of Bone Morphology Changes of Left Upper Extremity Bones

Generally, the muscles and bones of the dominant hand are more developed than those of the contralateral upper extremity, and the bony prominences at the muscle stops are also more developed [15, 16]. The background to this recognition is that the presence of continuous external mechanical stimulation is essential for maintaining bone morphology and strength [1, 2]. Therefore, when permanent motor nerve paralysis results in muscle paralysis and restriction of bone and joint movement, bone strength is reduced, and subsequently, bone morphology is changed. Prolonged paralysis of the left upper extremity of Mashiki 15 caused muscle atrophy, leading to disuse atrophy. Disuse atrophy is a change that progresses over a period of years. Especially in the growing skeleton, the presence of motor paralysis leads to significant changes in bone morphology. Since the left upper extremity of Mashiki 15 was significantly thinner than the right upper extremity, it is assumed that the motor paralysis occurred at a younger age. Takeuchi [17] found that bone growth inhibition occurred in the transverse direction of membranous ossification in a patient who died after being bedridden for 16 years from birth due to hydrocephalus. However, there was minor retardation of growth in the longitudinal direction of cartilaginous ossification. The growth of all three extremities, except for the left upper extremity, was comparable to that of an adult female, indicating that Mashiki 15 was not bedridden and could maintain a certain amount of activity.

The paralysis of the muscles of the left upper extremity resulted in the loss of external mechanical stimulation and the suppression of membranous ossification of the bone. However, Mashiki 15 survived by carrying out some activities with the help of the upper extremity.

The preservation of the epiphyses is worse on the left side than on the right side of the upper extremity bones of Mashiki 15. Generally, the epiphyses contain more cancellous bone, which is less well preserved than the cortical bone of the diaphysis. Furthermore, in the present case, the left upper extremity bones were atrophic compared to the right, which could make the cancellous bones even more fragile. Thus, the difference in the preservation of the epiphyses between the right and left sides could be explained.

### 4.2. Differential Diagnosis of Mashiki 15

Neurological problems are the first suspected cause of motor paralysis of the extremities. In Mashiki 15, bone growth was observed in three extremities except for the left upper extremity, so systemic diseases like muscular dystrophy and congenital skeletal dysplasia were excluded from the differential diagnosis.

Paralytic diseases of the motor nerves can be broadly divided into central and peripheral paralyses. Central paralysis is caused by disorders of the brain or spinal cord, both of which are often severe enough to be life-threatening. The most common causes of paralysis due to brain damage are cerebral palsy, head trauma, cerebral infarction, and intracerebral haemorrhage. Paralysis due to spinal cord disease is caused by traumatic spinal cord injury or spinal cord tumours. Central paralysis often affects the lower extremities, and the complications are often severe [18, 19]. Given the level of medical care and living conditions in ancient times, it is assumed that those who suffered severe complications in childhood would have found it difficult to survive into adulthood. Because Mashiki 15 survived into young adulthood, the possibility of central nervous system paralysis is minimal.

Peripheral nerve palsy, on the other hand, is often limited in extent to the nerves that are paralysed and occurs in one side of the upper or lower extremity. Thus, it is possible to live a long life with some disabilities and limitations in daily life. Peripheral nerve palsy can be caused by various factors, including peripheral nerve damage from trauma, permanent compression of peripheral nerves from neoplastic disease, or infectious diseases such as acute poliomyelitis. Particularly in paralysis limited to one upper extremity, the differential includes brachial plexus injury due to trauma, delivery palsy at birth, and acute poliomyelitis due to polio.

The Brachial plexus comprises the fifth, sixth, seventh, and eighth cervical ventral rami and the first thoracic ventral ramus. It innervates the muscles, joints, and skin of the upper extremity. The brachial plexus travels from medial to lateral, dividing into the root, trunk, division, and cord, while branching nerves innervate various upper extremity parts [20].

Brachial plexus injury can be caused by external forces from high-energy trauma, such as a fall while riding a motorcycle or during high-speed sports such as skiing. It can also be damaged directly by a puncture wound in the supraclavicular fossa or a bone fragment from a clavicle fracture. Accidents resulting in high-energy trauma are unlikely to have occurred in the period when Mashiki 15 lived. However, the possibility of injury due to a fall from a height cannot be ruled out. The brachial plexus stretching can also injure it during delivery due to the force exerted by the birthing manoeuvre to separate the head from the shoulder. Brachial plexus palsy due to delivery is referred to as delivery palsy. Approximately 10–30% of infants who suffer brachial plexus injury at birth will have residual neurological deficits and will present with permanent changes in upper extremity development and function if not adequately treated [21].

Brachial plexus palsy is classified according to the height and extent of injury into superior (the fifth and sixth ± seventh cervical roots), total (the fifth to eighth cervical root + the first thoracic root), inferior (the eighth cervical and the first thoracic root), and intermediate (the seventh cervical root) types [22–25]. In all types, severe and permanent paralysis results in disuse atrophy of the musculoskeletal system of the upper extremities. The superior type presents with motor deficits in the upper arm from the shoulder to the elbow and sensory deficits in the proximal lateral upper arm and lateral forearm. The total type presents with motor and sensory deficits in the entire arm from the shoulder to the hand. The inferior type causes paralysis of the forearm and hand, but it is often considered the total type at the time of injury, followed by incomplete recovery of the superior nerve roots, resulting in the inferior type [26]. In Mashiki 15, the left deltoid tuberosity was developed, while the forearm diaphysis was remarkably slender, suggesting that the lower nerve roots were paralysed compared to the upper roots. In ancient times, there was no surgical treatment as we know it today for brachial plexus injury, so there was no choice but to let the injury heal naturally.

Acute poliomyelitis is a viral disease that usually occurs in childhood and is transmitted by faecal excretion of the virus, which enters the body orally [27]. In most cases, the infection is subclinical and lifelong immunity is acquired, but paralysis occurs in 0.1–0.2% of cases. Of these, only a small percentage become permanently paralysed [28]. Paralysis is most common in the lower extremities, with unilateral lower extremity monoplegia being the most common. It is followed by unilateral upper extremity, bilateral lower extremities, and facial muscles [29, 30]. Of the 58 human remains excavated from the Mashiki-Azamabaru site, only Mashiki 15 showed pathological asymmetry of the extremity bones. Therefore, the possibility of a polio epidemic at this site is unknown. Ishida and Suzuki [31] reported on the morphology of modern human skeletons with disuse atrophy of the extremities caused by acute poliomyelitis in childhood. They found that the growth of the transverse diameter of the affected long bone was more inhibited than that of the long axis. In contrast, the bony development of the ligamentous attachments and epiphyses was relatively good. The degree of the longitudinal development of the left upper extremity of Mashiki 15 is unknown because the epiphyses did not remain. However, the possibility of polio cannot be ruled out because of the characteristic of weak bony development at the muscle attachments.

Besides neurological problems, the differential diagnosis for this skeleton is disuse atrophy due to early childhood trauma. There are no obvious signs of fracture in the remaining skeleton of the left upper extremity, but it is still possible that there has been severe trauma to the nonremaining part of the body, especially to the proximal humerus. Fractures of the proximal humerus in patients who are skeletally immature or approaching skeletal maturity are rare, but it is now recognised that nonsurgical treatment generally leads to good functional results [32, 33]. On the other hand, given the level of medical care and the environment in ancient times, it is possible that the fracture could have not been treated appropriately, leading to disuse atrophy. However, even if there had been severe trauma to the proximal humerus as described, significant atrophy of the left upper extremity skeleton, as in the present case, could not be explained by this because the distal forearm and hand were still movable if the nerves were not damaged. Likewise, if there had been severe trauma to the nonremaining left elbow joint and hand in early childhood, it is unlikely that the entire left upper extremity skeleton would have atrophied as much as it did in this case. This is because if the injury is more distal, the proximal skeleton can move somewhat. This implies the presence of an external mechanical stimulus, which should be able to maintain the morphology and strength of the skeleton.

### 4.3. Palaeopathological Reports of Bone Growth Disorder in the Unilateral Upper Extremity

There are several palaeopathological reports about the growth of unilateral upper extremity bones. Hershkovitz et al. [34] reported a right-side dominant asymmetry in a male human skeleton, Ohalo II, excavated from the Upper Palaeolithic Ohalo site in Israel and diagnosed it as an adult-onset Erb-Duchenne-type brachial plexus palsy of the left upper extremity. On the other hand, Trinkaus [35] reexamined Ohalo II based on a comparison with data from other human skeletons from the Upper Palaeolithic. Based on this comparison, it was concluded that the asymmetry of the upper extremity bones of Ohalo II was within the expected range for Upper Palaeolithic human remains and that there is no evidence for an upper extremity anomaly. Churchill and Formicola [36] reported bilateral differences in the upper extremity bones of an adult male skeleton labelled Barma Grande 2, excavated from an Upper Palaeolithic cave in Barzilossi, Liguria, Italy. The percentage asymmetry calculated for Barma Grande 2 as 100 × (right − left)/left was smaller than that for Mashiki 15. The authors suggest that the factors that produced the asymmetry in Barma Grande 2 developed after the skeleton had matured, as the asymmetry in the diaphysis was greater than that in the articular and muscular insertions.

Lieverse et al. [9] reported an adult male skeleton with severe bilateral upper extremity asymmetry, designated Shamanka II 29.1, from the early Neolithic cemetery of Shamanka II on the south coast of Lake Baikal, Siberia, Russia. The most striking asymmetry was between the bilateral humerus, ranging from 11.7% to 89.5%. In the diseased extremity, no structures of muscle attachment, including the deltoid tuberosity, were observed. Because the asymmetry extended over the entire upper extremity, the authors concluded that it reflected complete brachial palsy occurring before the arm skeleton matured. In the skeleton of Mashiki 15, the greatest degree of asymmetry was observed in the bilateral ulna, with a range of 46.2% to 75.8%. The presence of the left deltoid tubercle of Mashiki 15, which was absent in Shamanka II, suggests that the brachial plexus injury was not the complete total type but rather a pathology with incomplete recovery of at least the fifth cervical root from the total type.

## 5. Conclusion

Mashiki 15, a human skeleton from the middle to late Okinawa Shell Midden Period, was buried alone at the Mashiki-Azamabaru site in Okinawa Prefecture. The most likely disease of this asymmetry was the brachial plexus palsy, which was considered to have been caused by birth palsy, trauma, or acute poliomyelitis in childhood. The type of brachial plexus injury was not the total type, as the deltoid tubercle was observed, and it was assumed that the fifth cervical root was not originally injured or that it had recovered incompletely from the total type. Prolonged motor nerve paralysis results in disruption of the skeletal remodelling process, leading to impaired bone growth. Any paralytic disease would have taken years or longer to produce changes in bone tissue. Even in ancient times, when the medical and welfare environment was not as well developed as it is today, there was a strong fellowship and a mentally stable society that accepted the existence of individuals with long-term physical disabilities, such as in this case. The palaeopathological study of Mashiki 15 would provide an essential basis for the future interpretation and diagnosis of similar cases.

## Figures and Tables

**Figure 1:** The Mashiki-Azamabaru site located in Ginowan, Okinawa Prefecture, Japan.

**Figure 2:** (a) Photograph of Mashiki 15, a young adult human skeleton buried alone in the Mashiki-Azamabaru site. (b) Schematic diagram of the skeletal remains of Mashiki 15 in its buried condition. There was no artificiality in the continuity and layout of the excavated skeleton.

**Figure 3:** The remaining part of Mashiki 15. The shaded area is the residual part.

**Figure 4:** Anterior and right lateral views of the skull. The black arrow indicates the osteoma on the right external auditory canal.

**Figure 5:** (a) Comparison of both lower extremity bones. (b) Comparison of both upper extremity bones.

**Figure 6:** (a) Arrows indicate the deltoid tubercles of the bilateral humerus. (b) Cross-sectional images at the level of the distal quarter of the bilateral radius. (c) Cross-sectional images at the level of the middle of the bilateral ulna. A: anterior; P: posterior; R: right; L: left.

**Figure 7:** (a) Cross-sectional images of the bilateral humerus at the level of the minimum circumference measurement. (b) Cross-sectional images of the bilateral radius at the level of the minimum circumference measurement. (c) Cross-sectional images of the bilateral ulna at the level of the minimum circumference measurement. A: anterior; P: posterior; R: right; L: left.

**Table 1:** Measurements of upper and lower extremity bones belonging to Mashiki 15 and percentage asymmetry calculated as 100 × (maximum − minimum)/minimum. Martin numbers are given in parenthesis as appropriate.

	Left (mm)	Right (mm)	Percentage asymmetry
Humerus			
Maximum diameter of midshaft (M5)	13.8	21.2	53.6
Minimum diameter of midshaft (M6)	12	15.8	31.7
Least circumference of the shaft (M7)	42	59	40.5
Radius			
Maximum transverse shaft diameter (M4)	11.5	14.6	27.0
Minimum sagittal shaft diameter (M5)	7.3	10.7	46.6
Minimum circumference (M3)	28	38	35.7
Ulna			
Dorsoventral shaft diameter (M11)	8.4	13.5	60.7
Transverse shaft diameter (M12)	9.1	16	75.8
Least circumference (M3)	26	38	46.2
Femur			
Anterior-posterior diameter of the midshaft (M6)	25.4	24.9	2.0
Mediolateral diameter of the midshaft (M7)	20.0	20.5	2.5
Circumference of the midshaft (M8)	74	73	1.4
Tibia			
Sagittal diameter at the midshaft (M8)	26.2	26.5	1.2
Transverse diameter at the midshaft (M9)	18.7	19.3	3.2
Circumference of the midshaft (M10)	71	73	2.8

**Table 2:** Comparison of the Mashiki 15 left-side humerus, radius, ulna, femur, and tibia measurements to the adult mean value dimensions and those of children of the Ohtomo site. Martin numbers are given in parenthesis as appropriate.

	Mashiki 15		Ohtomo site								
			Male, left			Female, left			9-year-old	9-year-old	10-year-old
	Left	Right	Mean	SD	*N*	Mean	SD	*N*	Right	Right	Right
Humerus											
Maximum diameter of midshaft (M6)	13.8	21.2	23.44	1.54	34	20.95	1.7	20	14.3	15.5	16
Minimum diameter of midshaft (M7)	12	15.8	17.58	1.64	33	15.8	0.95	20	10.7	12.1	12.2
Least circumference of the shaft (M8)	42	59	64.52	3.33	33	57.58	2.77	19	39	44	44
Radius											
Maximum transverse shaft diameter (M5)	11.5	14.6	17.12	1.17	25	16.36	1.28	11	10.6	11.5	10.7
Minimum sagittal shaft diameter (M6)	7.3	10.7	12.36	0.81	25	11.18	0.4	11	7.5	8.4	7.9
Minimum circumference (M4)	28	38	44.67	2.15	15	40.44	2.88	9	28	30.5	29
Ulna											
Dorsoventral shaft diameter (M12)	8.4	13.5	15.04	0.92	26	12.83	1.27	11	7.8	8.4	—
Transverse shaft diameter (M13)	9.1	16	17.15	1.38	26	15.91	1.12	12	11.1	11.9	—
Least circumference (M4)	26	38	37.18	2.9	22	33.86	1.35	7	—	25	—
Femur											
Anterior-posterior diameter of the midshaft (M7)	25.4	24.9	28.61	2.71	41	25.23	1.39	30	—	19.3	20.7
Mediolateral diameter of the midshaft (M8)	20	20.5	26.43	1.65	42	25.2	1.73	30	—	17	15.8
Circumference of the midshaft (M9)	74	73	86.98	5.46	41	80.41	4.46	29	—	57	58
Tibia											
Sagittal diameter at the midshaft (M9)	26.2	26.5	30.95	2.13	43	27.63	2.16	24	—	21.2	20.1
Transverse diameter at the midshaft (M10)	18.7	19.3	21.35	1.66	43	19.65	1.13	26	—	16.3	15.4
Circumference of the midshaft (M11)	71	73	83.39	5.56	41	75.26	4.4	23	—	50	57

## Data Availability

The data used to support the findings of this study are included in the article.
